# The Potential Therapeutic Effect of Guanosine after Cortical Focal Ischemia in Rats

**DOI:** 10.1371/journal.pone.0090693

**Published:** 2014-02-28

**Authors:** Gisele Hansel, Denise Barbosa Ramos, Camila Aguilar Delgado, Débora Guerini Souza, Roberto Farina Almeida, Luis Valmor Portela, André Quincozes-Santos, Diogo Onofre Souza

**Affiliations:** Programa de Pós Graduação em Ciências Biológicas-Bioquímica, Departamento de Bioquímica, Instituto de Ciências Básicas da Saúde, Universidade Federal do Rio Grande do Sul, Porto Alegre, RS, Brazil; Albany Medical College, United States of America

## Abstract

**Background and Purpose:**

Stroke is a devastating disease. Both excitotoxicity and oxidative stress play important roles in ischemic brain injury, along with harmful impacts on ischemic cerebral tissue. As guanosine plays an important neuroprotective role in the central nervous system, the purpose of this study was to evaluate the neuroprotective effects of guanosine and putative cerebral events following the onset of permanent focal cerebral ischemia.

**Methods:**

Permanent focal cerebral ischemia was induced in rats by thermocoagulation. Guanosine was administered immediately, 1 h, 3 h and 6 h after surgery. Behavioral performance was evaluated by cylinder testing for a period of 15 days after surgery. Brain oxidative stress parameters, including levels of ROS/RNS, lipid peroxidation, antioxidant non-enzymatic levels (GSH, vitamin C) and enzymatic parameters (SOD expression and activity and CAT activity), as well as glutamatergic parameters (EAAC1, GLAST and GLT1, glutamine synthetase) were analyzed.

**Results:**

After 24 h, ischemic injury resulted in impaired function of the forelimb, caused brain infarct and increased lipid peroxidation. Treatment with guanosine restored these parameters. Oxidative stress markers were affected by ischemic insult, demonstrated by increased ROS/RNS levels, increased SOD expression with reduced SOD activity and decreased non-enzymatic (GSH and vitamin C) antioxidant defenses. Guanosine prevented increased ROS/RNS levels, decreased SOD activity, further increased SOD expression, increased CAT activity and restored vitamin C levels. Ischemia also affected glutamatergic parameters, illustrated by increased EAAC1 levels and decreased GLT1 levels; guanosine reversed the decreased GLT1 levels and did not affect the EAAC1 levels.

**Conclusion:**

The effects of brain ischemia were strongly attenuated by guanosine administration. The cellular mechanisms involved in redox and glutamatergic homeostasis, which were both affected by the ischemic insult, were also modulated by guanosine. These observations reveal that guanosine may represent a potential therapeutic agent in cerebral ischemia by preventing oxidative stress and excitotoxicity.

## Introduction

Ischemic stroke is the second most common cause of death and the major cause of disability worldwide [1]–[5]. According to the American Heart Association, someone has a stroke every 40 seconds, and stroke accounts for one of every 18 deaths in the United States [6]. The sudden reduction in blood flow leads to decreased oxygen and glucose supplies to the ischemic brain area, resulting in a failure of cellular bioenergetics. This condition triggers a series of events known as the ischemic cascade, during which the degree of damage is dependent on the affected area and length of blood flow blockage. Disruption of brain metabolism is clearly a key element in stroke, resulting in cellular damage and impairment of neurological functions [1], [2],[4], [5].

Both excitotoxicity and oxidative damage are ischemic events related to cerebral energy failure [1], [2], [4]. Due to energy depletion, excitatory amino acid transporters (EAATs), EAAT1/glutamate-aspartate transporter (GLAST) and EAAT2/glutamate transporter-1 (GLT1) in astrocytes and EAAT3/excitatory amino acid carrier 1 (EAAC1) in neurons [7], [8], responsible for glutamate uptake, are adversely affected, enabling high intracellular concentrations of glutamate to drive the transporters into reverse, releasing toxic amounts of the neurotransmitter into the synapse [7], [9]. The excessive glutamate levels in the synaptic cleft leads to overstimulation of glutamate receptors. This overstimulation initiates several molecular events that trigger a massive generation of free radical species and extensive cellular damage [1], [2],[4], [10].

Thus, the brain parenchyma undergoes dramatic changes in oxygen homeostasis, generating more free radical species that play important roles in ischemia and reperfusion injury [2],[4], [5], [11]–[13]. The central nervous system (CNS) has an efficient antioxidant defense system, including superoxide dismutase (SOD), catalase (CAT) and glutathione peroxidase (GPx), as well as scavenger molecules such as glutathione (GSH) and vitamin C. Despite the effectiveness of this system, the endogenous antioxidant capacity can be overwhelmed during cerebral ischemia, resulting in overproduction of free radicals including reactive oxygen species (ROS) and reactive nitrogen species (RNS), which have direct negative impacts on ischemic cerebral tissue [5] [11] [13] [14]. ROS/RNS trigger many cellular and molecular events, including protein oxidation/nitrosylation/nitration, lipid peroxidation and DNA damage, resulting in damage to macromolecules and consequent activation of signaling mechanisms that lead to cell death [2] [4] [5] [11] [13]. Thus, molecules with antioxidant activities are anticipated to have beneficial effects on brain ischemia.

It has been demonstrated that guanosine (GUO), a guanine-based purine, plays important roles in the CNS [15]–[23]. Endogenous GUO levels increase after 2 h of focal stroke and remain higher for 7 days [24]. This finding led to the investigation of the effects of exogenously administered GUO on stroke models. The data from *in vitro* models suggests that GUO protects against oxygen and glucose deprivation (OGD) [25]–[29], increases glutamate uptake in hypoxia-ischemia models [30], [31], and is neuroprotective against permanent and transient ischemic stroke [25], [32], [33]. In addition, GUO demonstrates antioxidant activity, protecting DNA from oxidative damage [34], [35], and modulates oxidative and nitrosative stress in neurotoxic models [36], [37]. Studies are pointing that GUO may exert its effects through modulation of mitogen-activated protein kinases (MAPKs) and phosphoinositide 3-kinase (PI3K) signaling pathways [27]–[29], however, the mechanisms of the protective effects of GUO are not fully understood yet.

As previous experimental studies have demonstrated that GUO acts as a neuroprotective agent against stroke and is able to modulate oxidative response and glutamatergic parameters [33], [35], [36], the objectives of this study are to investigate the potential neuroprotective role of GUO using a model of permanent focal cerebral ischemia. For that, the focus of this study is directed to explore the neural intracellular biochemical parameters as well as underlying neuroprotective mechanisms.

## Materials and Methods

### Animals

Adult male Wistar rats (90–100 days old, weighing 300–350 g) were maintained under controlled light and environmental conditions (12 h light/12 h dark cycle at a temperature of 22±2°C) with water and commercial food *ad libitum*. All experimental procedures were performed according to the NIH Guide for Care and Use of Laboratory Animals and the Brazilian Society for Neuroscience and Behavior (SBNeC) recommendations for Animal Care and were approved by the ethical committee from Federal University of Rio Grande do Sul (Process number: 19283). All efforts were made to minimize the number of animals used and to prevent suffering.

### Induction of Permanent Focal Ischemia

Ischemic lesion was induced by thermocoagulation of the blood in the pial vessels of the motor and sensorimotor cortices [38]. Briefly, the animals were anesthetized with ketamine hydrochloride (70 mg/kg, i.p.) and xylazine hydrochloride (10 mg/kg, i.p.) and placed in a stereotaxic apparatus. The skull was surgically exposed and a craniotomy was performed, exposing the left frontoparietal cortex (+2 to −6 mm A.P. and −2 to −4 mm M.L. from bregma), the motor and sensorimotor cortex regions [39]. Blood in the pial vessels was thermocoagulated transdurally by approximation of a hot probe to the Dura mater. The color of the blood vessels is normally light red, and the development of a dark red color was an indicator of complete thermocoagulation. After the procedure, the skin was sutured and body temperature was maintained at 37°C using a heating pad until recovery from the anesthesia.

### Drug Treatment

The animals were divided into four groups: Sham Saline (SS), Sham GUO (SG), Ischemia Saline (IS) and Ischemia GUO (IG). GUO (60 mg/Kg in NaCl 0.9%) was purchased from Sigma (St. Louis, MO, USA). The GUO dose was chosen based on a dose-response curve test of the beneficial effect of GUO administration, as evaluated by the spontaneous exploratory behavior of rodents (cylinder test) for 15 days. First, a study was conducted with a GUO pretreatment 30 min before induction of ischemia, along with administration of GUO at 1 h, 3 h and 6 h after induction of ischemia (**Figure 1A**). After this initial dose-range finding experiment, a dose-response curve for GUO was obtained, but instead of pretreatment with GUO, GUO was administered immediately after induction of ischemia. Thus, all groups received a 1 mL/kg intraperitoneal (i.p.) administration (saline or GUO) immediately, 1 h, 3 h and 6 h after surgery (**Figure 1B**). Based upon these results, it was administrated GUO (60 mg/kg i.p.) immediately, 1 h, 3 h and 6 h after surgery.

**Figure 1:** GUO dose-response curve. The beneficial effects of GUO were evaluated by a cylinder test. (**A**) Cylinder Test on 0, 1, 3, 7 and 15 days post-ischemia. GUO i.p. administration was performed 4 times (30 min before ischemia and 1 h, 3 h and 6 h after ischemia). *represents *P*<0.001 when comparing ischemia saline vs. sham saline and ^#^represents *P*<0.001 when comparing ischemia saline vs. ischemia GUO 30 mg/Kg. n = 9–10 per group. (**B**) Cylinder Test on 0, 1, 3, 7 and 15 days post-ischemia. GUO i.p. administration was performed 4 times (immediately, 1 h, 3 h and 6 h after ischemia). *represents *P*<0.001 when comparing ischemia saline vs. sham saline, ^#^represents *P*<0.01 when comparing ischemia saline vs. ischemia GUO 60 mg/Kg and ^&^represents *P*<0.01 when comparing ischemia saline vs. Ischemia GUO 120 mg/Kg. n = 9–13 per group.

### Cylinder Test

This test evaluates the spontaneous exploratory behavior of rodents [40], [41]. The cylinder test reveals forelimb preference when the animal rears to explore its environment by making forelimb contact with the cylinder walls. Animals were subjected to one trial on the pre-ischemic day. To prevent habituation to the cylinder, the number of movements recorded was limited to 20. The occurrences of sole use of the ipsilateral (to the lesion) or contralateral forelimb, or the simultaneous use of both forelimbs, were counted. The asymmetry score for each animal was calculated each day by the formula previously described [42]. For the dose-response curve experiments with GUO administration, animals were tested on 1, 3, 7 and 15 days post-ischemic injury. For all other experiments, the animals were tested 24 h after ischemia, before the biochemical experiments.

### Measurement of Infarct Volume

Twenty-four hours after surgery, animals were sacrificed, and the brains were rapidly removed from the skull and sectioned in the coronal plane at 2 mm of thickness, using a rat brain matrix (Insight LTDA, Ribeirão Preto, SP, Brazil). The slices were immersed for 30 min into 2% of 2,3,5-triphenyltetrazolium chloride (TTC) (Sigma, USA) solution at 37°C, followed by overnight fixation in 4% paraformaldehyde (Sigma, USA). The infarct volume was calculated by the formula: *Infarct volume  =  [measured infarct area × slice thickness (2 mm)]+[area of contralateral corresponding structure × slice thickness]–[area of ipsilateral corresponding structure × slice thickness]* [43] [44]. The brain slices were analyzed by Image J software (NIH, USA). The results are expressed as mm^3^.

### Tissue Processing

All neurochemical parameters were evaluated 24 h after the ischemic insult. The animals were decapitated under deep anesthesia, and the brains were removed from the skull and maintained at 4°C. In ischemic animals, the cortical tissue surrounding the ischemic lesion, located between the lesion and the cerebral longitudinal fissure (a piece measuring approximately 8 mm×2 mm), was dissected. This region was chosen because previous studies using this model pointed that it has characteristics similar to the penumbra. In sham animals, the same region was dissected [42] (**Figure 2**).

**Figure 2:** Schematic illustration of the ischemic lesion. Illustrations showing the region of the induced lesion (gray) and the analyzed region (dark gray) that were dissected for the experiments. The left frontoparietal cortex (+2 to −6 mm A.P. and −2 to −4 mm M.L. from bregma) was used.

For measurement of intracellular ROS levels, cortical slices (300 µm) were immediately incubated, and the experiment specimens were processed. For glutamine synthetase activity, the tissue was homogenized in a 150 mM KCl solution. For other oxidative stress assays, the tissue was homogenized in 20 mM sodium phosphate buffer, pH 7.4, containing 140 mM KCl. For Western Blot analysis, the tissue was homogenized using lysis solution [4% SDS, 2 mM EDTA, 50 mM Tris-HCl, pH 6.8], containing a protease and phosphatase inhibitors cocktail, and normalized with sample buffer [62.5 mM Tris-HCl, pH 6.8, 2% (w/v) SDS, 5% β-mercaptoethanol, 10% (v/v) glycerol, 0.002% (w/v) bromophenol blue]. All homogenates were frozen (at −80°C) until the biochemical measurements were conducted.

### Thiobarbituric Acid-reactive Substances (TBARS) Measurement

Lipid peroxidation can be evaluated by the TBARS assay [37], which evaluates the lipid damage via assay-based detection of malondialdehyde, the last product of lipid breakdown caused by oxidative stress. Briefly, homogenates (10 µL) were added to 20 µL of cold 10% trichloroacetic acid and 30 µL of 0.67% thiobarbituric acid in 7.1% sodium sulfate and boiled for 1 h. The mixture was cooled in water for 3 min. Afterwards, 40 µL of butyl alcohol were added, and then these samples were centrifuged at 5,000 *g* for 5 min. Pink-colored TBARS was determined in the resulting supernatants using a spectrophotometric microtiter plate reader set to read at 532 nm. A calibration curve was performed using 1,1,3,3-tetramethoxypropane. The data are expressed as nmol/mg of protein.

### Intracellular ROS Levels

DCFH oxidation was used to measure intracellular ROS production. DCFH-DA (2′-7′-dichlorofluorescein diacetate) is hydrolyzed by intracellular esterases to dichlorofluorescin (DCFH), which is trapped within the cell. This non-fluorescent molecule is then oxidized to fluorescent dichlorofluorescin (DCF) by the action of cellular oxidants. Cortical slices were treated with DCFH-DA (10 µM) for 30 min at 37°C. Following DCFH-DA exposure, the slices were placed into PBS with 0.2% Triton X-100. Fluorescence was measured in a plate reader (Spectra Max M5, Molecular Devices, USA) with excitation at 485 nm and emission at 520 nm [45]. The ROS production was calculated as fluorescence units per milligram protein (UF/mg) and then expressed as a percent of control.

### Nitric Oxide (NO) Levels

NO was determined by measurement of nitrite (a stable oxidation product of NO), based on the Griess reaction [46]. Briefly, homogenates were mixed with 25% trichloroacetic acid and centrifuged at 1,800 *g* for 10 min. The supernatant was immediately neutralized to pH 7.0 with 2 M potassium bicarbonate. NO_3_ was reduced to NO_2_ by nitrate reductase. Total NO_2_ was measured by a colorimetric assay at 540 nm. A standard curve was performed using sodium nitrate (0–80 µM). The results are expressed as µM of nitrite/mg of protein.

### Vitamin C Levels

Ascorbic acid (AscH^−^) was used to indicate vitamin C levels. Homogenates were centrifuged at 10,000 *g* for 2 min. Aliquots (50 µL) of the supernatant samples or AscH^−^ standards were placed in a 96-well plate, and 50 µL of the 4-hydroxy-2,2,6,6-tetramethylpiperidinyloxy (Tempol) stock solution (2.32 mM Tempol in acetate buffer) were added, and then these samples were incubated for 10 min at room temperature. While protecting the reaction from light, 21 µL of *o*-phenylenediamine (OPDA) solution (5.5 mM OPDA in acetate buffer) was added. Tempol promotes the oxidation of ascorbic acid to dehydroascorbic acid, which was measured by fluorescence detection (345 nm for excitation and a 425 nm for emission) in a Spectra Max GEMINI XPS plate reader (Molecular Devices, USA) [47]. The results were expressed as µM of AscH^−/^mg of protein.

### GSH Levels

GSH levels were assessed as previously described [48]. Briefly, homogenates were diluted in 10 volumes of 100 mM sodium phosphate buffer, pH 8.0, containing 5 mM EDTA, and the protein was precipitated with 1.7% meta-phosphoric acid. The supernatant was mixed with *o*-phthaldialdehyde (1 mg/mL methanol) and incubated at room temperature for 15 min. Fluorescence was measured using excitation and emission wavelengths of 350 and 420 nm, respectively. A calibration curve was performed with standard GSH solutions (0–500 µM). The GSH concentration was calculated as nmol/mg of protein.

### SOD Activity

SOD activity was determined using the RANSOD kit from Randox (Autrim, United Kingdom). This method is based on the formation of red formazan from the reaction of 2-(4-iodophenyl)-3-(4-nitrophenol)-5-phenyltetrazolium chloride and the superoxide radicals produced in the incubation medium from the xanthine and xanthine oxidase reaction system, which is assayed spectrophometrically at 505 nm. Inhibition of the produced chromogen is proportional to the activity of the SOD. The 50% inhibitory concentration is defined as one unit of SOD, and the specific activity is represented as U/mg of protein.

### CAT Activity

CAT activity was assayed as previously described [49]. The absorbance was measured in homogenized tissue by measuring the absorbance decrease at 240 nm in a reaction medium containing: 20 mM H_2_O_2_, 0.1% Triton X-100, 10 mM potassium phosphate buffer, pH 7.0, and 50 µg protein. One unit (U) of the enzyme is defined as 1 µmol of H_2_O_2_ consumed per minute. The results were expressed in U/mg of protein.

### Glutamine Synthetase (GS) Activity

The enzymatic assay was performed as previously described [50]. Briefly, homogenates (0.1 mL) were added to 0.1 mL of the reaction mixture containing: 10 mM MgCl_2_, 50 mM L-glutamate, 100 mM imidazole-HCl buffer (pH 7.4), 10 mM 2-mercaptoethanol, 50 mM hydroxylamine-HCl and 10 mM ATP, and incubated for 15 min at 37°C. The reaction was stopped by the addition of 0.4 mL of a solution containing 370 mM ferric chloride, 670 mM HCl, and 200 mM trichloroacetic acid. Samples were centrifuged at 1,000 *g* for 10 min, and the absorbance of the supernatant was measured at 530 nm and compared to absorbance generated by standard quantities of γ-glutamyl-hydroxamate treated with ferric chloride reagent. The results are expressed as µmol/h/mg of protein.

### Western Blot Analysis

Samples (20 µg protein/well) were subjected to SDS-polyacrylamide gel electrophoresis and transferred to a nitrocellulose membrane. Membranes were processed as follows: (1) blocking with 5% bovine serum albumin for 2 h; (2) incubation with primary antibody overnight [anti-SOD1, anti-EAAC1, anti-GLAST and anti-GLT1 (1∶1000) from Alpha Diagnostic (St. Antonio, TX, USA) and anti-β-actin (1∶5000) and anti-β-tubulin (1∶10000) from Santa Cruz Biotechnology (Santa Cruz, CA, USA)]; (3) incubation with peroxidase conjugated secondary antibody for 2 h; and, finally, (4) chemiluminescence (ECL kit) was detected using X-ray films. The films were scanned, and the bands were quantified using Image J software (NIH, USA). The results are expressed in percent of control levels.

### Protein Assay

Protein content was measured using Pierce BCA protein kit (Thermo Scientific, USA) with bovine serum albumin as the standard. The results are expressed as mg of protein.

### Statistical Analysis

The results are presented as the mean ± S.E.M. The cylinder test was analyzed with a repeated-measures analysis of variance (ANOVA), followed by Tukey’s post-hoc test. Infarct volume was analyzed using Student’s t-test. Oxidative stress assays and Western blots were statistically analyzed using two-way analysis of variance (ANOVA) followed by the Bonferroni’s post-hoc test. Correlations were analyzed by Pearson’s correlation. Probability values less than 0.05 were considered statistically significant. All analyses were performed using the Statistical Package for Social Sciences (SPSS) software version 15.0.

## Results

### GUO Treatment Partially Restored Function of the Impaired Forelimb, Reduced Brain Infarct Volume, and Prevented Lipid Damage in Brain Tissue

GUO treatment led to a partial recovery in the function of the impaired forelimb after 24 h of permanent focal cerebral ischemia, and the effect was maintained up to 15 days post-insult. No dysfunction of the forelimb was observed in the sham group (**Figure 3A**). Brain infarct volume analysis by TTC staining 24 h after ischemia showed tissue damage in the ischemic animals, visualized by pale stained-tissue (**Figure 3B**). GUO treatment significantly decreased the size of the area of tissue damage (**Figures 3B and 3C**). No tissue damage was observed in sham groups (**Figure 3B**). There was an increase in lipid damage in the ischemic group [ischemic effect: F_(1,32)_ = 28.8; *P*<0.0001], which was abolished by GUO treatment (**Figure 3D**).

**Figure 3:** GUO treatment improved forelimb function and reduced cerebral damage caused by ischemic insult. (**A**) Cylinder Test 24 h before and 24 h after ischemia; *represents *P*<0.001 when comparing ischemia saline (IS) vs. sham saline (SS) and sham GUO (SG); ^#^represents *P*<0.001 when comparing ischemia saline (IS) vs. ischemia GUO (IG); n = 10–15 per group. (**B**) Representative coronal brain sections (2 mm thick) stained with 2% TTC demonstrating infarction. Red-colored regions indicate a non-ischemic area, and pale-colored regions indicate the ischemic area. (**C**) Analysis of the cortical infarct volume measured by TTC staining, 24 h after cerebral ischemia; the data are expressed as mm^3^. *represents *P* = 0.012 with n = 8 per group. (**D**) Lipid peroxidation was measured by the TBARS method 24 h after ischemia. The data are expressed as nmol/mg of protein. ***represents *P*<0.001 with n = 7–11 per group.

### GUO Treatment Decreased ROS/RNS Levels and Modulated Important Antioxidant Defenses Following Permanent Focal Cerebral Ischemia

Twenty-four hours after ischemic insult, ROS [ischemic effect: F_(1,32)_ = 13.0; *P* = 0.0012] and NO [ischemic effect: F_(1,32)_ = 8.0; *P* = 0.008] levels increased in the ischemic group, and these effects were prevented by GUO treatment (**Figures 4A and 4B**).

**Figure 4:** ROS/RNS levels increased 24 h after ischemia, and GUO treatment prevent this effect. (**A**) Effects on ROS levels, measured by DCF fluorescence as described in the Materials and methods section. The data are expressed as percent of control (n = 7–11 per group). (**B**) Effects on NO levels expressed as µM/mg of protein (n = 7–11 per group). The production of NO levels was indirectly measured by the formation of nitrite, as described in the Materials and methods section. The results expressed as the mean ± S.E.M. **represents *P*<0.01; ***represents *P*<0.001.

Analysis of the non-enzymatic antioxidant molecules in the CNS demonstrated that ischemic insult decreased GSH levels from 290.6±8.5 to 249.4±14.6 nmol/mg of protein [ischemic effect: F_(1,31)_ = 16.1; *P = *0.0003] and that GUO treatment did not prevent this effect (**Figure 5A**). Additionally, vitamin C levels (**Figure 5B**) decreased significantly in the ischemic group [ischemic effect: F_(1,32)_ = 130.0; *P*<0.0001], and the GUO treatment partially restored these levels [treatment effect: F_(1,32)_ = 11.5; *P = *0.00018].

**Figure 5:** Analysis of non-enzymatic and enzymatic antioxidant defenses 24 h after the ischemia. (**A**) Effect on GSH levels, measured as described in the Materials and methods section. The data are expressed as nmol/mg of protein (n = 7–11 per group). (**B**) Effect on vitamin C levels measured as AscH^−^, measured as described in the Materials and methods section. The data are expressed as µM/mg of protein (n = 7–11 per group). (**C**) Effect of SOD expression, measured by western blot. The data were normalized by β-tubulin and are expressed as a percent of control (n- 6–9 per group). Effect on enzymatic antioxidant activities: (**D**) SOD activity and (**E**) CAT activity. The data are expressed as U/mg of protein (n = 7–11 per group). *indicates *P*<0.05, **indicates *P*<0.01 and ***indicates *P*<0.001.

Analysis of the antioxidant enzymes in the CNS suggests that GUO modulated the effects of ischemic injury. There was a large increase (5-fold) in SOD expression (**Figure 5C**) measured 24 h after the ischemic insult [ischemic effect: F_(1,24)_ = 144.3; *P*<0.0001] when compared to the sham group. Surprisingly, SOD activity did not demonstrate the same profile (**Figure 5D**); despite the presence of increased SOD expression, the SOD enzyme activity decreased in the ischemic group. GUO treatment following ischemia increased both SOD expression and activity. Although the ischemic insult did not affect CAT activity (**Figure 5E**), ischemic animals treated with GUO presented an increased CAT activity [treatment effect: F_(1,32)_ = 13,7; P = 0.008].

### GUO Modulated Glutamatergic Parameters Affected by the Ischemic Insult

When measured 24 h after ischemic injury, expression of the neuronal EAAC1 transporter (**Figure 6A**) increased in the ischemic group [ischemic effect: F_(1,26)_ = 13.0; *P = *0.0013], and GUO had no effect on this increase. The analysis of glial glutamatergic transporters GLAST and GLT1 showed a different profile. The ischemic insult did not affect GLAST expression (**Figure 6B**). However, GLT1 expression (**Figure 6C**) following the ischemic insult was significantly diminished [ischemic effect: F_(1,24)_ = 18.0; *P = *0.0003], and GUO treatment prevented this effect [treatment effect: F_(1,26)_ = 5.5; *P = *0.027].

**Figure 6:** Analysis of glutamatergic transporters by Western blot 24 (**A**) EAAC1 expression, (**B**) GLAST expression and (**C**) GLT1 expression measured by western blot. The data are expressed as a percent of control (n = 6–9 per group). The same membranes were blotted against β-tubulin to serve as a loading control. **indicates *P*<0.01 and ***indicates *P*<0.001.

The activity and expression of GS, the enzyme responsible for conversion of glutamate to glutamine in astrocytes, were evaluated 24 h after ischemia. GS protein expression was similar in all groups (**Figure 7A**). Interestingly, ischemic insult did not affect GS activity [ischemic effect: F_(1,50)_ = 3.6; *P = *0.062], but GUO treatment of the ischemic group resulted in increased GS activity (**Figure 7B**).

**Figure 7:** Effects of ischemia and GUO treatment on GS measured 24 (**A**) GS activity, measured by colorimetric method that evaluate the enzyme activity metabolizing glutamate (substrate) into glutamine (product), as described in the Materials and methods section. The data are expressed as µmol/h/mg of protein (n = 11–16 per group). (**B**) GS expression, measured by western blot analysis. The data were normalized by β-actin and are expressed as a percent of control (n = 6–9 per group). *indicates *P*<0.05.

### Correlation of Oxidative Stress Parameters and the Declining Function of the Impaired Forelimb

The data analysis was performed to investigate any potential correlation between the function of the impaired forelimb (symmetry score) and antioxidant scavenger (vitamin C) levels, reactive species (intracellular ROS) levels, and/or lipid damage (lipid peroxidation). There was a strong positive correlation of the symmetry score with vitamin C levels (**Figure 8A**; R^2^ = 0.72, *P*<0.0001), and there was a moderate negative correlation of the symmetry score with ROS levels (**Figure 8B**; R^2^ = 0.31, *P* = 0.008) and with lipid peroxidation (**Figure 8C**; R^2^ = 0.41, *P*<0.0001).

**Figure 8:** Correlation between oxidative stress parameters and forelimb function (symmetry score) measured 24 h after ischemia. (**A**) Positive correlation with vitamin C levels (AscH^−^). (**B**) Negative correlation with ROS levels. (**C**) Negative correlation with lipid peroxidation.

## Discussion

Acute ischemic stroke causes sudden impairment of blood circulation in a brain area, resulting in a failure of bioenergetics and cellular damage [1], [2], [4]. Despite considerable advances in the understanding of the pathophysiology of cerebral ischemia, therapeutic options for stroke are still limited. Previous studies have demonstrated beneficial effects of GUO against ischemic insult. GUO was able to recovery the sensorimotor function and reduce the cerebral infarct volume in both, permanent and transient Middle Cerebral Artery Occlusion (MCAO) [25] [32], [33]. Corroborating with these data, the present study found that GUO treatment caused a significant recovery in the function of impaired forelimb, and this effect was maintained up to 15 days post-insult (last measurement), and also significantly reduced the cerebral infarct volume. Moreover, GUO treatment significantly abolished the increase in lipid peroxidation caused by ischemia. Thus, GUO treatment was able to restore clinical sensorimotor function, decreased the associated morphological brain damage and abolished the neural cell membrane damage. These results demonstrate an effective neuroprotective role of GUO against ischemic insult to the brain.

The mechanisms of neuroprotective strategies against cerebral ischemia may target biochemical alterations involved in cellular damage and/or improve hemostatic and vascular systems involved in collateral blood flow. As the precise GUO neuroprotective mechanisms are unclear, this study aimed to search for putative intracellular biochemical parameters in neural cells involved in this neuroprotection. Here, it was demonstrated for the first time that GUO treatment modulated important parameters related to both the oxidative stress response (redox homeostasis system) and the glutamatergic system after an *in vivo* ischemic event.

Free radicals play an essential role in maintaining the physiological condition of the body. Because the CNS has a high oxidative metabolism rate, brain cells are especially vulnerable to free radical damage during ischemia [4], [5], [11]. Defense against free radicals is provided by a number of antioxidant enzymes, including SOD, CAT and GPx. SOD converts O_2_^−^ to H_2_O_2_, whereas CAT and GPx convert H_2_O_2_ to H_2_O, thus removing ROS. These enzymes are coupled with other non-enzymatic antioxidants, such as GSH and vitamin C, responsible for reducing both ROS and RNS levels [51]–[53]. During an ischemic event, there is a massive production of ROS (generated by the mitochondrial respiratory chain and NADPH oxidase) and RNS (generated by the combination of NOS and superoxide, forming the peroxynitrite) [54] [55] that depletes intracellular brain GSH and vitamin C levels [55]–[57]. Despite increased expression of antioxidant enzymes during ischemic injury, there is an impairment of their activities, which implies a severe state of oxidative stress and enhanced lipid peroxidation rates [11], [13]. Here, the ischemic insult increased SOD expression and decreased SOD activity; GUO treatment increased SOD expression and completely reestablished SOD activity. Studies have shown that overexpression of SOD in transgenic mice resulted in a reduction of infarction volume and better neurological outcomes after ischemia [51], [58], [59]. The increased CAT activity in the ischemic animals treated with GUO could be a beneficial response designed to remove H_2_O_2_. In this context, modulation of the expression and activity of SOD and the CAT activity by GUO may indicate that the neuroprotective effects of GUO are associated with attenuation of oxidative stress, consequently decreasing free radical levels [11], [51], [59].

Mounting evidence suggests that radical scavengers mediate protective effects following cerebral ischemia [60] [61]. Studies have shown vitamin C is neuroprotective during ischemia, decreasing infarct volume, and this effect is likely related to scavenging for reactive species [56], [61]. In the current study, ischemic insult decreased the levels of the non-enzymatic scavenger compounds GSH and vitamin C; although GUO treatment was not able to reverse the decreased GSH levels, GUO treatment did reverse the decreased vitamin C levels, increasing the presence of this non-enzymatic scavenger in the ischemic environment. Therefore, the neuroprotection of GUO in cerebral ischemia could be related to its enhancement of endogenous antioxidant capacity and inhibition of reactive species production, thereby mitigating the brain damage caused by reactive species production resulting from ischemia.

Glutamate excitotoxicity has long been recognized to play a key role in the pathophysiology of cerebral ischemia. Ischemia impairs glutamate uptake by EAATs, contributing to toxic amounts of the neurotransmitter into the synapse [7] [9]. These events result in overstimulation of glutamatergic receptors and activation of intracellular pathways that lead to cell death [1], [2], [62]. Therefore, glutamate uptake activity is closely linked to ischemic events. GLAST and GLT1 are primarily expressed by astrocytes, which also express the enzyme GS to convert glutamate to glutamine, which is then recycled to glutamate into neurons. The connected activities of these proteins contribute to maintaining the extracellular glutamate concentration below toxic levels. EAAC1, on the other hand, is predominantly expressed in neurons [7]. The transport activities of EAAC1, GLAST and GLT1 are inhibited by oxidants via a direct action on the transporter proteins, reducing their activities [10], [63]. Herein, ischemic insult decreased GLT1 expression (the major astrocytic EAAT), effect reversed by GUO, and increased the neuronal EAAC1 expression, measured 24 h after ischemia. Although ischemia did not modify GS expression, its activity increased with GUO treatment after the insult. Thus, in the ischemic group, GUO potentially increased both the glutamate uptake and its intracellular conversion to glutamine. These effects may have increased removal of glutamate from the synaptic cleft in the surrounding brain area subjected to the ischemic insult. The function of EAAC1 in the brain has not been fully established. EAAC1 is a neuronal glutamate and cysteine transporter, involved in the regulation of synaptic glutamate uptake and responsible for uptake of cysteine and glutamate, precursors of GSH [8] [64] [65]. In this study, EAAC1 expression significantly increased 24 h after ischemia; it could be hypothesized that this increase is an endogenous protective mechanism in response to ischemic insult. Importantly, GUO treatment increased EAAC1 expression.

The correlation between the functional recovery of animals and the capacity for administration of GUO to abolish the decreased vitamin C levels, the increased ROS and RNS levels, and the increase in lipid peroxidation, demonstrates that these parameters are active participants in the pathogenesis of ischemia and the neuroprotective effects of GUO. Additionally, the recovery of essential functions of the glutamatergic system (including glutamate uptake and its metabolism) following GUO administration suggests that this is another important factor in the attenuation the tissue damage. Thus, although the mechanisms by which GUO acts are not fully known, it was demonstrated that GUO modulated maintenance of the cellular redox environment and the glutamatergic system following ischemic injury in rodents. Overall, our work represents an important contribution to the knowledge regarding the putative neuroprotective mechanisms of GUO in cerebral ischemia models. However, due to limitations of our model of brain ischemia, further studies in other robust models, such as MCAO, are necessary to evaluate the global relevance of GUO neuroprotection against cerebral stroke.
